# Polyetherketoneketone Mesh for Alveolar Bone Augmentation: Geometric Parameter Design and Finite Element Analysis

**DOI:** 10.1155/2023/8487380

**Published:** 2023-01-31

**Authors:** Xiaowen Hao, Wei Wang, Chenxi Wang, Jianmin Han, Yu Zhang

**Affiliations:** ^1^Department of Implantology, Peking University School and Hospital of Stomatology, Beijing 100081, China; ^2^National Clinical Research Center for Oral Diseases, National Engineering Laboratory for Digital and Material Technology of Stomatology, Beijing Key Laboratory of Digital Stomatology, Research Center of Engineering and Technology for Computerized Dentistry Ministry of Health, NMPA Key Laboratory for Dental Materials, Beijing 100081, China; ^3^Urumql DW Innovation InfoTech Co.,Ltd., Urumqi, Xinjiang 830013, China; ^4^Department of Dental Materials, Peking University School and Hospital of Stomatology, Beijing 100081, China

## Abstract

**Objective:**

To evaluate the mechanical properties of porous polyetherketoneketone (PEKK) meshes with different thicknesses, pore sizes, and porosities through finite element analysis to provide an optimal PEKK design for alveolar bone augmentation in the posterior mandibular region.

**Methods:**

A three-dimensional evaluation model of severe alveolar bone defects in the mandibular posterior was constructed based on cone beam computerized tomography (CBCT) data. Then, PEKK meshes with different structural designs were obtained. Two key parameters were set with different values: five levels of thickness (0.2 mm, 0.3 mm, 0.4 mm, 0.5 mm, and 0.6 mm) and three levels of pore size (1 mm, 2 mm, and 3 mm) with a corresponding porosity of 19.18%–42.67%. A 100 N physiological force was simultaneously loaded by finite element analysis (FEA), and the deformation and stress data were outputted for further analysis.

**Results:**

The deformation and stress of the PEKK meshes are negatively correlated with the changes in thickness and positively correlated with the changes in pore size. The FEA results show that the maximum deformation, equivalent stress, and maximum principal stress of the PEKK meshes are 0.168 mm–0.478 mm, 49.243 MPa–124.890 MPa, and 31.549 MPa–104.200 MPa, respectively. The PEKK mesh group with a thickness of 0.2 mm, pore size of 3 mm, and porosity of 42.67% is in danger of plastic deformation or even fracture during use.

**Conclusion:**

According to the FEA results, the PEKK meshes with larger thicknesses and smaller pore sizes and porosities behave better. In consideration of reducing soft tissue stimulation and promoting bone regeneration, an ultrathin porous PEKK mesh with a pore size of no more than 3 mm, porosity of no more than 42.67%, and thickness of 0.2 mm can be used clinically to meet the mechanical performance requirements of the guided bone regeneration (GBR) structure.

## 1. Introduction

To reestablish dentition function, dental implant surgery is a widely accepted treatment with predictable effects [1] and has become the main choice for patients. As stable bone volume has been considered a prerequisite for successful implant surgery [2], severe periodontal disease, trauma, and tumors often cause severe atrophy or large alveolar bone defects, which are the main challenges for the current implantology based on osseointegration. Guided bone regeneration (GBR), one of the most commonly used methods, has clinically reliable outcomes regarding alveolar bone augmentation [3]. When performing GBR surgery for the bone augmentation of severe bone defects, a barrier membrane scaffold with a certain mechanical strength is often required to maintain the stability of the osteogenic space. The rigidity of the titanium-reinforced expended polytetrafluorethylene (e-PTFE) membrane ensures its stability during use, and this type of membrane is widely used for bone augmentation. However, the manual bending and trimming of the 2D scaffold material is required during traditional surgery, and bent shapes are often difficult to fit into complex anatomical structures. The time-consuming shaping process and possible sharp edges also increase the risk of soft tissue dehiscence and infection [4], predisposing patients to varying degrees of bone augmentation failure [5].

With the progress in materials science and digital technology, individualized barrier membrane scaffolds that can accurately fit the shape of the reconstructed alveolar ridge can be obtained, enabling restoration-oriented bone augmentation surgery and the design of implant restoration. The individualized scaffold materials that can be digitally designed include metals, such as titanium, and high-performance polymer materials. In recent years, high-performance polymer materials with excellent physicochemical properties and good machinability have become a popular research topic in the application of individualized barrier membrane scaffolds. Among these materials, polyaryletherketone (PAEK) is a stand-out thermoplastic composite due to its ultrahigh mechanical properties and chemical resistance, and its main component, polyetheretherketone (PEEK), exhibits excellent mechanical properties and biological activity and is widely used in the biomedicine field. Recently, there have been clinical studies on the application of individualized PEEK in alveolar bone defect reconstruction, and satisfactory clinical results have been obtained [6, 7]. A recent finite element analysis (FEA) showed that under the load of occlusal force, it is possible for a porous PEEK mesh with a thickness of 0.6 mm to remain relatively stable and have abilities to maintain space and form new bone similar to those of titanium mesh [8].

Space maintenance ability and stability are the key functions of the GBR membrane scaffold, and mechanical properties are one of its primary reference indicators. However, due to the lack of relevant research on the structural design and mechanical properties of individualized PEEK, there is not yet a clear understanding of the mechanical properties of PEEK materials. In addition, the reported PEEK obtained by computer-assisted design/computer-assisted manufacturing (CAD/CAM) with redundant thickness not only increases the difficulty of the clinical operation but also may affect the healing and osteogenesis of the bone graft due to a potentially insufficient blood supply. Moreover, the FEA results suggest that ultrathin PAEK materials have the potential to be barrier membrane scaffolds, and their optimal design needs to be urgently studied. Not only do pore size and porosity have profound impacts on biological properties, such as bone ingrowth and cell and nutrient transport [9], but also thickness is a key design parameter that affects the mechanical properties of barrier membrane scaffolds. Therefore, for their common clinical applications, it is necessary to explore their geometric parameter design to obtain better clinical operability while meeting the biomechanical property requirements.

Polyetherketoneketone (PEKK) is a polyarylether polymer similar to PEEK. Compared with those of PEEK materials, the superior mechanical properties and antibacterial properties of PEKK materials endow them with greater potential as barrier membrane scaffold materials. In the process of evaluating the mechanical properties of PEKK meshes by traditional mechanical property tests, we found that 3D printing PEKK technology is not yet mature, with high raw material requirements and a high cost. Additionally, the precision of the test PEKK sample obtained by computer numerical control (CNC) machining is poor and cannot meet the experimental design requirements. Finally, we chose the FEA method, which has unique advantages for studying biomechanical behavior, to evaluate the mechanical properties of individualized PEKK meshes.

In this study, we selected severe bone defects in the posterior mandibular area, which is the most common in clinical practice, as the mechanics evaluation model for bone defect reconstruction. We evaluated the mechanical properties of PEKK meshes with different thicknesses, pore sizes, and porosities under simulated physiological loads through FEA to provide a reference for the geometric parameter design of individualized PEKK structures for alveolar bone augmentation in the posterior mandibular area.

## 2. Materials and Methods

### 2.1. Geometric Reconstruction

A 3D geometrical model was constructed based on cone-beam computerized tomography (CBCT) data from a patient who had severe alveolar bone defects in the mandibular posterior area (Figure 1). The authors confirmed that the patient provided informed consent for data collection. The CBCT images (slice thickness 0.2 mm and pixel size 0.200 mm) were input as digital imaging and communications in medicine (DICOM) files for 3D model reconstruction into Mimics 20.0 software (Materialise NV, Belgium). For further noise reduction and smoothing, a standard tessellation language (STL) file was input into Geomagic Studio 2014 software (3D System, USA) and NX 1911 software (Siemens, Germany). A 3D model of the periodontal ligament with a thickness of 0.2 mm was obtained by expanding outward from the tooth surface, and the mandibular bone defect model was shifted inward by 1.5 mm as the cancellous bone model. The periodontal ligament and cancellous bone models were obtained by Boolean operation, and based on the virtual bone augmentation morphology (Figure 2), the PEKK mesh design was obtained. The height of the bone graft was 3 mm at the bottom of the dental crown restoration, and the width of the bone graft was at least 10 mm. The specifications of the titanium screws were designed to be 1.4 mm in diameter and 7 mm in length, and the adjusted positions of the titanium screws were at least 2 mm away from the adjacent teeth, mental foramen, and mandibular canal [10]. Finally, a virtual mandible bone augmentation model was obtained, which contained cortical bone, teeth, periodontal ligament, cancellous bone, bone graft, PEKK mesh, and titanium screws.

### 2.2. Finite Element Modeling

The special FE software ANSYS Workbench 2019 (ANSYS, USA) was used to calculate the models, which were defined as isotropic, homogeneous, continuous elastic materials. We designed and built fifteen 3D-FE models of the PEKK mesh with thicknesses of 0.2 mm, 0.3 mm, 0.4 mm, 0.5 mm, or 0.6 mm and a pore size of 1.0 mm, 2.0 mm, or 3.0 mm (Table 1).

To achieve greater simulation accuracy, the interface between the PEKK mesh with the cortical bone and the graft bone was set to be in frictional contact with a friction coefficient of 0.2 [11]. The junctions between other models were set to be rigidly connected, such as the connection between the PEKK mesh with titanium screws. According to the literature, Table 2 lists the material properties of the PEKK, cortical bone, periodontal ligament, bone graft, teeth, cancellous bone, and titanium.

The ascending mandibular ramus, the lower edge of the mandible, and the median symphysis were set as the boundaries to limit the movement of the model. In the axial direction, we applied a functional loading force of 100 N to the model [17] (Figure 3). Then, the deformation and stress data of the PEKK mesh were output for follow-up analysis.

## 3. Results

### 3.1. Establishment of the Mechanics Evaluation Model

By establishing a mechanical evaluation model based on virtual bone augmentation through advanced digital imaging technology combined with a variety of software, we successfully built fifteen 3D-FE individualized PEKK mesh models under strict boundary conditions (Figure 4). The models can simulate the mechanical performance of the barrier membrane and have good geometric similarity.

### 3.2. 3D-FEA Results of the PEKK Meshes

Taking the deformation of two groups of PEKK meshes with a pore size of 1 mm and a thickness of 0.6 mm and a pore size of 3 mm and a thickness of 0.2 mm as examples (Figure 5), the displacement from the lingual side to the alveolar ridge and then to the buccal side increases gradually, and the maximum displacement occurs when the alveolar crest migrates to the buccal bone plate.  Figure 6 shows the overall deformation distribution of 15 PEKK mesh groups, ranging from 0.168 mm to 0.478 mm.

The equivalent stress of different PEKK meshes ranges from 49.243 MPa to 124.89 MPa (Figure 7), and the maximum principal stress ranges from 31.549 MPa to 104.2 MPa (Figure 8). The two figures show that the distribution trend of the equivalent stress is the same as that of the maximum principal stress, and the maximum stress is concentrated at the turning point of the buccal alveolar ridge. The group with the largest maximum principal stress of 104.2 MPa, which is very close to the extreme tensile strength, is the group of PEKK meshes with a pore size of 3 mm, thickness of 0.2 mm, and porosity of 42.67%, suggesting that this PEKK mesh group may suffer plastic deformation or even fracture during use.

### 3.3. Influences of Thickness and Pore Size on the PEKK Meshes

The FEA results show that with decreasing thickness (0.6 mm–0.2 mm) and increasing pore size and porosity (1 mm–3 mm; 19.18–42.67%), the maximum deformation and stress values of the PEKK meshes increase (Figure 9). These changes are negatively correlated with the changes in thickness and positively correlated with the changes in pore size.

Moreover, by using multiple linear regression analysis, the deformation, equivalent stress, and maximum principal stress of the PEKK meshes are used as dependent variables to analyze the corresponding influences of the thickness and pore size (Tables 3–5). The regression models have a statistical significance (*P* < 0.05), which means that both thickness and pore size significantly affect the deformation and stress distributions of the PEKK meshes. The *F* change of the multiple regression analysis model of the deformation of PEKK is 152.149, and the adjusted *R* squared value is 0.956. The *F* change of the multiple regression analysis model of the equivalent stress of PEKK is 42.155, and the adjusted *R* squared value is 0.855. The *F* change of the multiple regression analysis model of the maximum principal stress of PEKK is 36.777, and the adjusted *R* squared value is 0.836.

## 4. Discussion

PAEK is a linear aromatic polyetherketone with a stable para-aromatic ring structure that results in superior mechanical properties and chemical resistance as a thermoplastic composite [13]. Moreover, its good biocompatibility has made it an alternative material for titanium in the field of orthopedics and a promising restorative material in stomatology, and PAEK materials have been applied in removable partial dentures, full-crown restorations, implant abutments, root posts, and cores [18–20]. Both PEEK and PEKK have aromatic ring structures, but their ratios of ether groups and ketone groups are different. Compared with PEEK, PEKK not only exhibits superior mechanical properties in terms of flexural, tensile, and compressive strength [21] but also its elastic modulus is closer to that of the bone tissue, and it has better antibacterial properties [20]. Therefore, in terms of mechanical properties and biological activities, PEKK is more suitable as a barrier membrane scaffold material than PEEK. However, the individualized PEKK structure design and application is still lacking and determining how to obtain an optimal scaffold structure design while meeting biomechanical performance requirements is crucial for its clinical application.

It is known that as design parameters, the thickness, pore size, and porosity of barrier membrane scaffolds significantly affect their mechanical properties, but the effects of these factors on clinical applications are complex and even contradictory in some cases [9, 22]. For example, increasing membrane thickness increases membrane stability but reduces the clinical management and volume of new bone; increasing pore size and porosity may enhance the efficiency of bone regeneration but substantially reduce membrane stiffness and strength. Therefore, the ideal PEKK scaffold should achieve better clinical operability on the basis of ensuring space maintenance. Among the methods for evaluating the mechanical properties of materials, the standard mechanical properties test is the most common and effective method, including tensile, compression, bending, and fatigue tests. Since Friedenberg first applied the finite element method to the medical field in 1969, with the development of computer technology and related software, the FEA has become a very effective analysis tool in the oral biomechanics field [23]. Therefore, because the existing methods of additive manufacturing and CNC machining cannot produce a test sample that meets experimental design requirements, 3D-FEA was used to investigate the stress distribution of PEKK meshes between the bone graft interfaces in this study, aiming at efficiently and quickly finding the optimal structure and providing a reference for clinical application. Our study takes full advantage of the structural advantages of FEA and reduces the dependence on a large number of human or animal experiments. A mechanical evaluation model for alveolar bone augmentation with good geometric similarity and biosimulation was successfully established.

PEKK is a new type of polymer material, and there is still a lack of preliminary clinical and experimental data relevant to its use as a barrier membrane scaffold. Therefore, when designing the thickness of PEKK, we refer to the titanium and PEEK meshes that have been clinically used. Under most circumstances, a thickness of 0.2 mm is enough for titanium mesh application [24], and another study reported that a 0.6 mm thick PEEK mesh was sufficient to maintain relative stability [8]. Therefore, considering that the mechanical properties of PEKK are between those of titanium and PEEK, this study set a thickness range from 0.2 to 0.6 mm to explore the mechanical properties of PEKK meshes. Moreover, the pore size of the barrier membrane scaffolds directly affects their mechanical strength, and their porous structures also affect vascularization and bone ingrowth. On the premise of ensuring mechanical properties, high porosity and large pore size tend to be selected to enhance bone regeneration. At present, the pore size of commercially available titanium meshes is usually at the millimeter level (usually 1–3 mm), which is why the author selected the pore size range from 1 to 3 mm. For the assignment of load force, considering that the Chinese usual bite force (UBF) is 100–150 N, the bone graft area does not directly bear the bite force but generally bears light pressure from food, tooth brushing, or chewing when speaking and swallowing that would not exceed the average bite force of the normal dentition. Finally, we set the 100 N physiological load force as the limit value of the PEKK's compressive capacity for the simulation.

According to the FEA results, with increasing mesh pore size and porosity (1–3 mm; 42.67–19.18%) and decreasing thickness (0.6–0.2 mm), there was a decrease in the mechanical behavior of the PEKK mesh. Furthermore, the thickness had a greater effect on the deformation and maximum principal stress than pore size, but the effect of pore size on the equivalent stress was greater than that of the thickness. All 15 groups of PEKK meshes showed good space maintenance ability under a 100 N physiological loading force; the maximum deformation was 0.478 mm, and the degree of displacement did not show the adverse effect of maintaining the osteogenic space, indicating that PEKK can remain relatively stable when used as a barrier membrane scaffold. The equivalent stress, also known as the von Mises stress, is related to the yield strength of the material; the maximum principal stress, also known as the tensile stress, is related to the tensile strength of the material. According to the literature [13, 25–27], the tensile strength of PEKK is approximately 102 MPa–115 MPa, which is much smaller than its compressive strength of 172 MPa–246 MPa and yield strength of 175 MPa. Since the edge of the PEKK mesh was fixed by titanium screws, when the stress was transmitted to the lateral displacement of the buccal and lingual, it was transformed into tensile stress. Therefore, the force leading to the breakage of the PEKK mesh should be tensile stress, and the broken site should be located at the turning point of the buccal and lingual sides, as the good toughness of PEKK may provide a certain buffer for compression in the alveolar ridge area. The group of PEKK meshes with a thickness of 0.2 mm, diameter of 3 mm, and porosity of 42.67% may be in danger of plastic deformation or even fracture during use, which is detrimental to the bone augmentation process. The maximum principal stress of the remaining groups ranged from 31.549 MPa to 72.91 MPa, which is far less than the tensile strength of PEKK, indicating that there is no danger of fracture during use.

Our study has its inevitable limitations as an FEA study. The loading condition was simplified to a single vertical loading force, but in clinical practice, the motor force of muscles such as the buccal muscles acting in the bone graft area after tension reduction and suture cannot be ignored. Therefore, it is necessary to further establish the masticatory muscle system and design different working conditions under clinical conditions to simulate the oral and jaw systems more realistically, such as alveolar bone defects in different regions, different stress angles, or placing implants simultaneously according to patient needs. Furthermore, since the finite element method is a computer numerical simulation, there are other limitations: changes in temperature, pH, load incidence, and fatigue are not taken into consideration, and the material is assumed to be homogeneous, linear, and free of defects. As a preclinical study of PEKK materials, the results of this study are limited to evaluating the feasibility of PEKK as a barrier membrane scaffold. Therefore, further animal experiments and clinical studies are needed to verify the real biomechanical and osteogenic performance of the PEKK mesh used for alveolar bone augmentation.

## 5. Conclusion

Our study successfully constructed a mechanical evaluation model with high simulation and good geometric similarity for alveolar bone defect reconstruction, which takes full advantage of the structural benefits of FEA and is also applicable for other GBR barrier membrane scaffold materials, such as polymers and metals. In addition, this is the first attempt at studying the biomechanics of individualized PEKK scaffolds. From a biomechanics perspective, this study provides a new option for the use of individualized barrier membrane scaffolds and provides a reference for the optimal design of PEKK as a barrier membrane scaffold material. The FEA results showed that the thickness, pore size, and porosity, as geometric parameters for the structural design of the PEKK mesh, are closely related to biomechanical performance. Within the range of FEA results, the larger the thickness and smaller the pore size and porosity are, the better the performance of the PEKK meshes, and PEKK has great potential for clinical application in terms of biomechanical properties. Considering that a barrier membrane should minimize soft tissue stimulation and maximize tissue integration functions, under the precondition of meeting the needs of alveolar bone defect reconstruction, ultrathin porous PEKK meshes with a 0.2 mm thickness, pore size of not more than 3 mm, and porosity of not more than 42.67% are preferred for clinical practice.

## Figures and Tables

**Figure 1:** CBCT screenshot and 3D reconstruction of severe bone defects in the posterior mandibular area.

**Figure 2:** Steps involved in the individualized PEKK mesh design. (a) Virtual implants; (b) virtual bone augmentation; (c) formation of bone graft and PEKK shell; (d) assembly of PEKK mesh, titanium screws, and bone graft; (e) adjustment of model position; (f) model of PEKK mesh.

**Figure 3:** (a) Range of functional loading force. (b) The arrow indicates the direction of force, and the blue area represents the border.

**Figure 4:** 3D-FE model of the PEKK mesh with different pore sizes: (a) pore size of 1 mm; (b) pore size of 2 mm; (c) pore size of 3 mm.

**Figure 5:** (a) Deformation of the PEKK mesh with a thickness of 0.6 mm and a pore size of 1 mm; (b) deformation of the PEKK mesh with a thickness of 0.2 mm and a pore size of 3 mm.

**Figure 6:** Deformation distributions of PEKK meshes with different thicknesses: (a) 0.2 mm. (b) 0.3 mm. (c) 0.4 mm. (d) 0.5 mm. (e) 0.6 mm.

**Figure 7:** Equivalent stress distributions of PEKK meshes with different thicknesses: (a) 0.2 mm. (b) 0.3 mm. (c) 0.4 mm. (d) 0.5 mm. (e) 0.6 mm.

**Figure 8:** Maximum principal stress distributions of PEKK meshes with different thicknesses: (a) 0.2 mm. (b) 0.3 mm. (c) 0.4 mm. (d) 0.5 mm. (e) 0.6 mm.

**Figure 9:** Relationship between the deformation (a), equivalent stress (b), and maximum principal stress (c) and the thickness and pore size of the PEKK meshes.

**Table 1:** Design parameters of the PEKK mesh.

Thickness (mm)	Porosity (%)		
	Pore size = 1 mm	Pore size = 2 mm	Pore size = 3 mm
0.2	19.56	34.31	42.67
0.3	19.40	33.95	42.18
0.4	19.27	33.79	41.98
0.5	19.19	33.62	41.72
0.6	19.18	33.54	41.61

**Table 2:** Material properties of model materials.

Materials	Young's modulus (MPa)	Poisson's ratio
PEKK	5100 [12–14]	0.40
Cortical bone	13700 [13, 14]	0.30
Cancellous bone	1370 [12–14]	0.30
Teeth	18600 [15]	0.31
Periodontal ligament	69 [15]	0.45
Bone graft	10 [16]	0.30
Titanium	110000 [10, 12, 13, 15]	0.30

**Table 3:** Multiple regression model of the deformation of the PEKK meshes.

	Unstandardized B	Coefficients std. error	Standardized coefficient beta^1^	Sig	95.0% confidence interval for B	
					Lower bound	Upper bound
(Constant)	0.411	0.019		<0.05	0.370	0.451
Pore size	0.046	0.006	0.442	<0.05	0.034	0.059
Thickness	−0.531	0.034	−0.876	<0.05	−0.065	−0.457

^1^The beta is the standardized regression coefficient, which is used to compare the absolute effect or absolute contribution between the coefficients. The larger the beta value is, the greater the absolute effect or absolute contribution. All beta values in the tables have the same meaning.

**Table 4:** Multiple regression model of the equivalent stress of the PEKK meshes.

	Unstandardized B	Coefficients std. error	Standardized coefficient beta	Sig	95.0% confidence interval for B	
					Lower bound	Upper bound
(Constant)	70.353	8.019		<0.05	52.882	87.824
Pore size	18.248	2.536	0.733	<0.05	12.724	23.773
Thickness	−83.484	14.640	−0.581	<0.05	−115.382	−51.587

**Table 5:** Multiple regression model of the maximum principal stress of the PEKK meshes.

	Unstandardized B	Coefficients std. error	Standardized coefficient beta	Sig	95.0% confidence interval for B	
					Lower bound	Upper bound
(Constant)	73.752	7.791		<0.05	56.776	90.728
Pore size	10.528	2.464	0.462	<0.05	5.160	15.896
Thickness	−105.779	14.225	−0.804	<0.05	−136.772	−74.785

## Data Availability

The data analyzed in this study are available from the corresponding author upon request.
